# A Topic Recognition Method of News Text Based on Word Embedding Enhancement

**DOI:** 10.1155/2022/4582480

**Published:** 2022-02-16

**Authors:** Qiming Du, Nan Li, Wenfu Liu, Daozhu Sun, Shudan Yang, Feng Yue

**Affiliations:** State Key Laboratory of Mathematical Engineering and Advanced Computing, Zhengzhou 450001, China

## Abstract

Topic recognition technology has been commonly applied to identify different categories of news topics from the vast amount of web information, which has a wide application prospect in the field of online public opinion monitoring, news recommendation, and so on. However, it is very challenging to effectively utilize key feature information such as syntax and semantics in the text to improve topic recognition accuracy. Some researchers proposed to combine the topic model with the word embedding model, whose results had shown that this approach could enrich text representation and benefit natural language processing downstream tasks. However, for the topic recognition problem of news texts, there is currently no standard way of combining topic model and word embedding model. Besides, some existing similar approaches were more complex and did not consider the fusion between topic distribution of different granularity and word embedding information. Therefore, this paper proposes a novel text representation method based on word embedding enhancement and further forms a full-process topic recognition framework for news text. In contrast to traditional topic recognition methods, this framework is designed to use the probabilistic topic model LDA, the word embedding models Word2vec and Glove to fully extract and integrate the topic distribution, semantic knowledge, and syntactic relationship of the text, and then use popular classifiers to automatically recognize the topic categories of news based on the obtained text representation vectors. As a result, the proposed framework can take advantage of the relationship between document and topic and the context information, which improves the expressive ability and reduces the dimensionality. Based on the two benchmark datasets of 20NewsGroup and BBC News, the experimental results verify the effectiveness and superiority of the proposed method based on word embedding enhancement for the news topic recognition problem.

## 1. Introduction

With the rapid development of information technology, people have been accustomed to obtaining various information from the Internet. These platforms, such as news websites and social media, enable us to know what is happening around the world whenever and wherever possible. However, under the current wave of information explosion, people are generally faced with the problem of having to spend much time and energy to find target information. Therefore, there is an urgent need to introduce topic recognition technology to identify news topics from texts, especially to identify different categories of news topics with different granularity to help enterprises or individuals quickly identify, extract, and analyze key information from the vast array of texts.

In recent years, topic recognition technology has become a research hotspot in the field of natural language processing (NLP). And, we notice that it has been widely used in online public opinion monitoring, news recommendation, search engine optimization, and other fields. During the classic topic recognition process, the text representation layer is responsible for converting texts into feature vectors that computers can understand and it is expected to minimize information loss, which is actually the foundation of the whole task [1]. As a matter of fact, the online news text is an important knowledge carrier, which has the characteristics of complex structures, wide sources, and huge volumes. In view of this situation, it is very challenging to effectively utilize key feature information such as syntax and semantics in the text to improve topic recognition accuracy.

From the 1970s to the present, text representation methods have undergone an evolution from shallow semantic to deep semantic. The traditional text representation model can be traced back to the Boolean Model method, which can efficiently process large-scale data while having the disadvantage of lacking semantic information. The emergence of the Vector Space Model (VSM) alleviates the problem of lacking semantic information to a certain extent, but high-dimensional sparsity and computational complexity are the major drawbacks. To explore the potential features of the text, researchers introduced probabilistic topic models, Latent Dirichlet Allocation (LDA) [2] and Biterm Topic Model (BTM) [3], which are suitable for long text topic modeling and short text topic modeling, respectively. The topic models have a solid theoretical foundation and they can make use of a limited number of hidden topics to realize low dimensional vector representation. The above is a review of the development of shallow semantic representation of text. In recent years, word embedding technology is developing rapidly, which brings more solutions to the NLP field. As one of the classic word embedding models, Word2vec [4] provides two training methods: Continuous Bag-of-Words (CBOW) and Skip-Gram (SG). During the training process, it adds multiple optimization methods (e.g., hierarchical softmax and subsampling) to reduce the computational complexity. Glove [5] is another one of the classic word embedding models, which can make better use of the common features of certain words to enrich the semantic information of word vectors and speed up the training process.

In terms of the design principles, the topic model such as LDA uses statistical inference methods to automatically discover the hidden patterns in a large-scale corpus. Based on this type of model, the text can be mapped to a low dimensional latent semantic space from the document-word matrix. The whole process has nothing to do with the language category and belongs to an unsupervised way. At the same time, the result is better interpretable [6]. However, the LDA model is based on the assumption of the Bag-of-Words (BOW) model, which naturally retains the shortcomings of this type of model, i.e., it ignores the semantic information between words [7]. With the word embedding model such as Word2vec, we can obtain a distributed dense vector to represent the text. Many studies have proved that such models based on *distributional hypothesis of linguistics* [8] can mine the semantic information contained in the text. The distributed dense vector representation is beneficial for downstream NLP tasks [9]. From the perspective of text mining, the above two models both achieve word-level clustering, but Word2vec is based on context, while LDA is based on implicit topics. From a more detailed perspective, we can think that Word2vec focuses more on co-occurrence information (fine-grained) of word and context, namely, semantic and syntactic information, while LDA focuses on the co-occurrence information (coarse-grained) of document and word, namely, document-topic information at a higher level. To some extent, these two models form a different but complementary relationship.

Based on the above analysis, this paper proposes a conjecture that the effective combination of topic model and word embedding model can enrich the text representation and benefit NLP downstream tasks. In recent years, some work has been carried out around this idea. Wang et al. [7] proposed to vectorize the high-probability word subset in each topic with Word2vec and LDA to obtain the topic vector, and then measured the Euclidean distance between the topic vector and the word embedding vector of each document as the new representation. Moody [10] proposed Lda2vec, which introduces LDA based on Word2vec to construct an unsupervised text representation that produces coherent topics. Zhou et al. [11] tried to combine the word embedding model, Term Frequency-Inverse Document Frequency (TF-IDF), and LDA, which had a better effect on the short text classification task. Peinelt et al. [12] proposed a simple framework tBERT, which combines topic model and Bidirectional Encoder Representations from Transformers (BERT) for semantic similarity prediction. Experiments show that this method can improve the accuracy on a series of semantic similarity prediction datasets.

However, due to the differences in target tasks, the updating of text representation models, and other factors, we can see that there is no standard framework for combining topic information and word embedding representation at present. For the topic recognition of news text, existing methods have been explored to improve the accuracy of recognition based on the above conjecture, but there are still some shortcomings. On the one hand, the model complexity is increased at the expense of time. On the other hand, the topic distribution of word or document reflects topic information in different granularities [13], so the fusion between topic distribution of different granularity and word embedding information is not considered.

In response to the above limitations, we propose a novel text representation method and form a full-process topic recognition framework for news text. In practice, this paper proposes to add word embedding vector as auxiliary information on the basis of LDA, and construct two kinds of text representations combined with topic information of different granularities: document-level topic distribution and document embedding (DTE) and word-level topic distribution and document embedding (WTE). Furthermore, we apply the two representations into the feature extraction layer in the proposed framework. The results show that this framework can make better use of the relationship between the document and the topic and the context information, which improves the expression ability and topic recognition accuracy. More specifically, our contributions are summarized as follows:

1. A text representation method based on word embedding enhancement is proposed. Considering the lack of semantics in the LDA topic model, and the word embedding models Word2vec and Glove have a good ability to capture semantic information, we tried to fuse the two types of models. Based on the topic distribution at document level and word level, two vector concatenation strategies were designed to incorporate more semantic information into the text representation.
2. A topic recognition framework for news text is proposed. The framework mainly includes three modules: preprocessing layer, feature extraction layer, and topic recognition layer. The preprocessing layer is responsible for performing necessary data cleaning, and the feature extraction layer is the concrete implementation of the proposed text representation method with different vector concatenation strategies. And, the topic recognition layer uses two popular classifiers: Support Vector Machine (SVM) and Logistic Regression (LR). The entire framework involves technologies such as BOW, LDA, word embedding, machine learning, and so on.
3. In this paper, several similar methods were selected as the baselines. Based on the two benchmark datasets of 20NewsGroup and BBC News, we conducted a comprehensive evaluation. The experimental results show that the performance of the proposed method is better than the baselines for news topic recognition.

The rest of the paper is organized as follows: Section 2 surveys and analyzes related work.  Section 3 describes the definition of related symbols and concepts.  Section 4 focuses on the description of the text representation method based on word embedding enhancement and the news topic recognition framework proposed in this paper.  Section 5 provides the details of experiments and further analysis. Finally, Section 6 gives the conclusion and the future research directions.

## 2. Related Work

### 2.1. Topic Detection and Tracking (TDT)

TDT is a kind of information processing technology oriented to text mining, which aims to monitor the information flow to realize the automatic recognition and classification of massive text data. At the same time, it can also detect hot events in specific fields, and merge the new text into a topic cluster by topic clustering, which can be used to track the progress of hot topics in large dynamic data.

Traditional TDT model mostly uses representation methods such as BOW and the topic model. Then, it uses text classification or clustering methods to perform topic recognition based on the obtained text vector representation. Obviously, the quality of the text representation largely lays the foundation of the topic recognition results, and the text classification or clustering models are also closely related to the accuracy and efficiency of the results. A lot of work has been carried out on these two aspects: Yan et al. [14] tried to improve TF-IDF and proposed the TF-IWF-IDF representation method. Compared with TF-IDF, this model incorporates semantic and contextual information. Huang et al. [15] proposed to combine LDA and Signal-pass for topic detection, which effectively improves the accuracy of topic detection. There are also some researches on TDT around the improvement of classification or clustering algorithms. Wan et al. [16] proposed a clustering algorithm RADBSCAN with relational awareness based on DBSCAN. This algorithm can determine the number of topics according to the dataset itself, and the topic recognition effect is better. Dai et al. [17] proposed an improved agglomerative hierarchical clustering method for topic detection, and it also can achieve topic tracking by adding the weight of feature terms in news titles during the similarity calculation process.

### 2.2. Text Representation

As an important research direction, the text representation plays a fundamental role in the NLP field. And, how to better represent text semantics to solve the practical applications is a problem under constant exploration. The classical methods can be traced back to the one-hot encoding, which belongs to the BOW model in essence. Then, the research focus has experienced the evolution from the topic model to the word embedding model [18]. Especially, with the development of deep learning technology and NLP, the word embedding model has gradually become a popular and effective method. Moreover, it has also been a hot topic in academia and industry in recent years.

#### 2.2.1. BOW

As the most basic text representation method, the BOW [19] separates the whole text with words as the basic unit of dimension. However, this method faces the problem of dimensional explosion and data sparsity. In response to high-dimensional issues, scholars propose evaluation indicators such as document frequency, mutual information (MI) [20], and information gain (IG) [21] for feature selection. For data sparsity, some methods about feature weight calculation have been proposed such as the classic TF-IDF. The core idea of TF-IDF is to count the appearance frequency of the word TF and the inverse document frequency IDF as the feature representation of the document. However, BOW and the classic TF-IDF method have a common problem of ignoring the semantic information of words [22].

#### 2.2.2. Topic Model

To further improve the quality of text representation, researchers try to explore the potential features. The Latent Semantic Indexing model (LSA) [23] uses the matrix decomposition method to realize the mapping from word vector space to semantic vector space, which solves the problem that traditional vector space models cannot deal with synonymy or polysemy. The probabilistic Latent Semantic Analysis (pLSA) [24] proposes a probability generation model to replace matrix decomposition and uses Expectation Maximization (EM) algorithm to estimate the parameters, which alleviates the interpretability problem of LSA to a certain extent. Latent Dirichlet Allocation (LDA) [25] is a three-layer Bayesian probability model, which contains a three-layer structure of documents, topics, and words. In LDA, each document can be represented as a topic distribution vector containing semantic information. The main value lies in: (1) This model implements the structuring of document, which also achieves the effect of dimensionality reduction compared with the BOW model; (2) This model completes document clustering and vocabulary clustering. Moreover, it realizes the abstract analysis of text information and reveals the semantic content implicit in the text. Thus, LDA is widely used in topic recognition problems [26–28].

#### 2.2.3. Word Embedding Model

In recent years, the rapid development of deep learning has opened up a new direction for the development of text representation [29]. In 2013, Mikolov et al. proposed the Word2vec model, which is a toolkit that allows seamless training and use of pre-trained embeddings. This model uses local sliding window, negative sampling, and other technologies, which bring new ideas to the industry. In 2014, Pennington et al. proposed another popular model Glove. This model makes full use of the co-occurrence matrix with global information and only trains the nonzero elements instead of the whole sparse matrix, which enriches the semantic information of the word vector and speeds up the training speed. Based on the pre-trained word embedding model, we can get the representation of words or characters in the text, and then obtain the representation of the entire text through operations such as convolution, pooling, and weighted summation [30]. Among them, the simplest method is to perform an average pooling operation on the word vectors.

However, it is also noteworthy that some more excellent models have been proposed, such as Embedding from Language Models (ELMo) [31], Generative Pre-Training Model (GPT) [32], and Bidirectional Encoder Representations from Transformers (BERT) [33]. After trained on a large corpus, they can capture more semantic information. However, their complexity is higher and they require stricter experimental conditions (GPU acceleration, memory capacity, etc.). For example, when operating on a document of length *N*, the complexity of Glove and BERT is *O*(*N*) and *O*(*N*^2^*H*), respectively, where *H* represents the maximum number of neurons in the hidden layer. Besides, BERT also limits the input length of the text sequence, and news text is usually long text data, which may lead to the loss of global information related to the task. Considering the complexity and recognition quality, this paper attempts to integrate the word embedding models, Word2vec, Glove, and topic model LDA to improve the quality of text representation. By integrating the advantages of each model, the new text representation includes not only the relationship between the document and topic but also the contextual relationship. Based on the new representation method, we design corresponding comparative experiments to verify the effectiveness of the proposed topic recognition framework.

## 3. Description of Symbols and Concepts

As shown in Table 1, the symbols involved in this paper are described in detail. For convenience in introducing the proposed text representation method and topic recognition framework, we also define some concepts in this section.

**Definition 1 .**

Word.

A word is the smallest unit in a document, where *T*_*i*_^*n*^ means that the element is the *n*th word in the *i*th document.

**Definition 2 .**

Document.

In this paper, a news document *D*_*i*_ is essentially sequences of words and can be described as *D*_*i*_=(*T*_*i*_^1^, *T*_*i*_^2^,…, *T*_*i*_^*n*^).

**Definition 3 .**

Corpus.

In this paper, a corpus *C* is essentially a collection of news documents, which can be denoted as *C*=(*D*_1_, *D*_2_,…, *D*_*m*_).

**Definition 4 .**

Topic distribution based on the LDA model.

Compared with traditional feature engineering, LDA has more advantages in text representation [11]. Assume that there are *ℵ* hidden topics in *m* documents, and all words *V* in the documents will also have a corresponding probability value for each topic, where *Z*=(*Z*_1_, *Z*_2_,…, *Z*_*ℵ*_) and *V*=(*T*_1_, *T*_2_,…, *T*_*n*_). As shown in Figure 1, we use an intuitive way to distinguish the document-topic distribution from topic-word distribution in the LDA model.

## 4. Methods

### 4.1. Text Representation Method Based on Word Embedding Enhancement

Based on the conjecture that “the effective combination of topic model and word embedding model can enrich the text representation” (refer to Section 1), this paper proposes to add word embedding vectors as auxiliary information on the basis of LDA topic model. In addition, Narayan et al. [13] proposed that the topic distribution of word reflects the topic information of the word itself and contains certain local context information, while the document-level topic distribution reflects the overall topic information of the document and contains global context information. Inspired by this, two text representation models of different granularities based on word embedding enhancement are designed, which are shown in Figure 2.

#### 4.1.1. Document-Level Topic Distribution and Document Embedding (DTE)

Based on the corpus *C*, the topic model TM can be obtained by training the LDA model. In addition, EM can also be obtained by training the word embedding model. For topic model, each document represents a probability distribution formed by some topics. Therefore, input the tokens contained in document *D*_*i*_ into TM, and the topic distribution of the document DTD_*i*_ can be obtained:

(1) $$\begin{array}{c} {\text{DTD}}_{i}=\text{TM}\left[T_{i}^{1},T_{i}^{2},\ldots ,T_{i}^{n}\right], \end{array}$$

where DTD_*i*_ ∈ *R*^*τ*^, |*D*_*i*_|=*n*, which shows that there are *n* words in document *D*_*i*_, and the document-level topic distribution DTD_*i*_ is a *τ*-dimensional vector. For document *D*_*i*_, the static representation of the included tokens can be easily obtained, and the word embedding of *D*_*i*_ is represented as

(2) $$\begin{array}{c} {\text{WE}}_{i}=\frac{\sum_{j=1}^{n}\text{EM}\left(T_{i}^{j}\right)}{n}, \end{array}$$

where *WE*_*i*_ ∈ *R*^*φ*^. Similar to the method in literature [12], the final target representation vector *DTE*_*i*_ is obtained by combining document-level topic representation and document embedding representation:

(3) $$\begin{array}{c} {\text{DTE}}_{i}=\left[{\text{DTD}}_{i}⊕{\text{WE}}_{i}\right]\in R^{\tau +\varphi }. \end{array}$$

#### 4.1.2. Word-Level Topic Distribution and Document Embedding (WTE)

For topic model, the topic-word distribution information can be obtained when training TM, which can be regarded as *ℵ* × *n* probability distribution matrix, where *ℵ* denotes the number of hidden topics and *n* denotes the number of words. After transposing, we can get the topic distribution of each word. For any token *T*_*i*_^*j*^ in *D*_*i*_, the word-level topic distribution *WTD*_*i*_ is calculated as follows:

(4) $$\begin{array}{c} {\text{WTD}}_{i}=\frac{\sum_{j=1}^{n}\text{TM}\left(T_{i}^{j}\right)}{n}, \end{array}$$

where WTD_*i*_, TM(*T*_*i*_^*j*^) ∈ *R*^*τ*^, which denotes that the topic distribution dimension of *T*_*i*_^*j*^ is *τ*, and the word-level topic distribution WTD_*i*_ is also a *τ*-dimensional vector. Similarly, the final representation vector *WTE*_*i*_ for document is obtained by concatenating the word-level topic representation and the document embedding representation:

(5) $$\begin{array}{c} {\text{WTE}}_{i}=\left[{\text{WTD}}_{i}⊕WE_{i}\right]\in R^{\tau +\varphi }. \end{array}$$

### 4.2. News Topic Recognition Framework

As shown in Figure 3, the whole framework mainly includes three submodules: (1) Text preprocessing layer, which is mainly responsible for performing necessary data cleaning such as removing stop words and low-frequency words. (2) Feature extraction layer. Based on the preprocessed text data, the topic model LDA and word embedding models, Word2vec and Glove, are used to extract feature information, and then obtain the text vector representation. (3) Topic recognition layer. This layer is mainly a classifier and aims at assigning a given news document to the most appropriate category.

#### 4.2.1. Preprocessing

Data processing is an important concept in many domains of scientific research [34,35]. In the NLP field, text data preprocessing plays an important role, which often determines the difficulty of training a model and the quality of the final results. There are many kinds of news data in the Internet, which have the characteristics of multi-source and heterogeneous. Thus, we need to do some preprocessing work to remove the interference information and retain as much important information as possible. In general, there is a large amount of noise information in the source data, so some necessary steps are often taken to remove it, which mainly includes removing punctuation, removing words that do not consist entirely of alphabetic characters, removing stop words, and so on. In addition, there are some words with a certain amount of information that appear less frequently in the text data. When they are put into the model for training, their existence often adds noise and reduces the quality of the model. Correspondingly, we will filter some low-frequency words. Finally, we will also remove short texts to improve the learning effect of the model on most of the distribution features of the text data.

#### 4.2.2. Feature Extraction

Within the whole framework, the feature extraction layer plays a pivotal role in transforming texts into vector representations with semantic information. And, the output of this layer largely determines the quality of the subsequent NLP tasks. Considering the complexity of the representation method and the recognition quality (refer to Section 2.2), the feature extraction layer will implement the proposed two text representations with different granularities based on Word2vec, Glove, and LDA. By incorporating the strengths of each model, the new text representation contains the relationship between the document and the topic and the context information, which demonstrates a stronger ability in feature extracting.

#### 4.2.3. Classifiers

To further utilize the obtained text representation to complete the topic recognition task, this framework will use two excellent classifiers: LR and SVM.

LR is a classic classification model. From a mathematical point of view, the model can be considered as adding a sigmoid function mapping on the basis of linear regression, which can improve the nonlinear capability. In more detail, the final goal of LR is to find the best plane to make the data linearly separable, while the nonlinear mapping reduces the weight of the points far away from the classification plane, and relatively increases the weight of the most relevant data points. Relatively speaking, LR is simple, easy to parallelize, and can be explained strongly, so it is often used to solve the binary classification problem in reality. The common solving methods of LR include stochastic gradient descent, Newton's method, etc. The cost function is a logarithmic loss function, which is generally expressed as follows:

(6) $$\begin{array}{c} J\left(\theta \right)=-\frac{1}{m}\overset{m}{\underset{i=1}{\sum }}\left(y_{i}\log\;h_{\theta }\left(x_{i}\right)+\left(1-y_{i}\right)\log\left(1-h_{\theta }\left(x_{i}\right)\right)\right)+\frac{\lambda }{2m}\sum_{j=1}^{n}\theta_{j}^{2}, \end{array}$$

where *h*_*θ*_(*x*_*i*_)=*θ*^*T*^*x*_*i*_+*b*. The part after “+” is a regularization term, which helps to alleviate the model's overfitting.

SVM is a generalized linear classifier that uses supervised learning to perform binary classification on data, whose final goal is to find the best classification hyperplane and ensure the maximum geometric interval. In the process of finding the decision boundary, SVM only considers the support vector, which is the local point near the classification surface. And, the ordinary samples other than the support vector will not participate in the final hyperplane decision. Therefore, the dependence on the number of training samples is greatly reduced, and the training efficiency is improved. In addition, for samples that are linearly inseparable in a finite-dimensional vector space, the appearance of kernel functions such as Gaussian, Laplace RBF, and Sigmoid realize the nonlinear separability of SVM. Generally speaking, the cost function of the SVM can be expressed as follows:

(7) $$\begin{array}{c} J\left(\theta \right)=\overset{m}{\underset{i=1}{\sum }}{\left(1-y_{i}h_{\theta }\left(x_{i}\right)\right)}_{+}+\lambda \sum_{j=1}^{n}\theta_{j}^{2}. \end{array}$$

The content within the whole bracket with “+” index is the hinge loss function, which has the following meaning:

(8) $$\begin{array}{c} {\left(1-y_{i}h_{\theta }\left(x_{i}\right)\right)}_{+}=\left\{\begin{array}{cc} 1-y_{i}h_{\theta }\left(x_{i}\right), & 1-y_{i}h_{\theta }\left(x_{i}\right)>0,\\ 0, & 1-y_{i}h_{\theta }\left(x_{i}\right)\leq 0. \end{array}\right.. \end{array}$$

## 5. Experiments and Discussion

In this section, all experiments are performed on a PowerEdge T640 tower server with Intel Xeon Gold 6238 processor, 128 GB DDR4 RDIMM memory, NVIDIA GeForce RTX 2080Ti. And, the software environment is CentOS 7.6, *Python* 3.7.7.

### 5.1. Data Preprocessing and Analysis

According to the task requirements, two commonly used News text datasets 20NewsGroup (https://scikit-learn.org/0.19/datasets/twenty_newsgroups.html) and BBC News (https://mlg.ucd.ie/datasets/bbc.html) are selected in this paper. These text data are all from the real world and marked with topic category tags.

#### 5.1.1. Overview of Datasets

20NewsGroup contains about 18,000 news articles, which can be classified into 20 news group collections. From the perspective of topic category tags, some groups have similar topics (such as talk.politics.guns and talk.politics.mideast which are related to guns and Middle East issues in the political field). Thus, it adds a certain degree of difficulty to topic recognition.  Table 2 gives a general description of the 20NewsGroup, where Len represents the average length of the topic news collection, and Size represents the number of documents in the corresponding collection. The overall distribution is relatively uniform.

Table 3 gives a general description of the BBC news dataset [36], which contains about 2225 news articles and covers five subject areas of technology, business, sports, entertainment, and politics. Note that the texts are all from the real BBC News website.

#### 5.1.2. Preprocessing and Parameter Settings

20NewsGroup and BBC News are both English text datasets, so we do not need to consider word segmentation for them. Besides, we will make use of some existing methods for preprocessing [37,38]. With the NLTK library in *Python*, we firstly filter out the common stop words, punctuations, numbers, and words with a total frequency of less than 3 in the document from the original text, then build and encode dictionaries based on the words.

After preprocessing, we input the text corpus into the topic recognition framework for model training. In order to make full use of the computing power of the server, the *LdaMulticore* training method in the GenSim library is called during LDA training. The parameters are set as *chunkSize* = 200, *passes* = 50, *workers* = 31, and the rest are the default values. When training Word2vec (https://github.com/PanJinquan/nlp-learning-tutorials/tree/master/word2vec), the training was carried out based on the CBOW model, with *iter* = 8 and *sg* = 0. When training Glove (https://github.com/stanfordnlp/GloVe), the parameters are set as *verbose* = 2. *memory* = 4.0, *vocab_min_count* = 5, *max_iter* = 15, *window_size* = 15, *binary* = 2, *num_threads* = 24, and *x_*max = 10. In addition, it is necessary to point out that the target output vector dimension is a scalar, and the specific value can be changed as needed. When calculating the vector representation of the target word, the word embedding model may encounter the OOV (out of vocabulary) problem. In this case, we will generate a vector of values between (0,1) in a specific dimension as the embedding representation of the word.

In this paper, we use LR and SVM to evaluate the effect of topic recognition. Both of these classifiers have detailed implementations in sklearn. To our best knowledge, the common methods for solving LR's loss function include *newton-cg*, *sag*, *lbfgs*, *liblinear*, and *saga*. After a lot of experiments, we chose to use *lbfgs* to solve the problem, with *max_iter* set to 100 and *C* set to 1.0. Regarding SVM, the kernel functions that can be used include *linear*, *poly*, *rbf*, *sigmoid*, and *precomputed*. After testing, we finally choose *linear*, with *C* set to 1 and *gamma* set to 1. For the purpose of enhancing the credibility of the experimental results, the parameters of the classifier are kept unchanged when compared with other models. Besides, the 5-fold cross validation method is adopted during the experiments.

### 5.2. Evaluation Indicators

#### 5.2.1. Topic Model

Macroscopically speaking, the topic model is a statistical model used to discover abstract topics in a series of documents. In the proposed topic recognition framework, the quality of the LDA model is closely related to the final topic recognition effect. Here, we will give relevant evaluation indicators.

Artificial topic quality judgment methods require a lot of manpower and material resources, and the emergence of those simulated artificial evaluation methods has brought new ideas to researchers. Among them, perplexity is a common topic model evaluation method [2]. In short, perplexity is to use probability to calculate the performance of a topic model on the test set. The higher the perplexity is, the more uncertain the topic model is to the document. Specifically, given a topic distribution *Z*, the formula for calculating the confusion degree of the trained topic model on the test set is as follows:

(9) $$\begin{array}{c} \text{perplexity}\left(C_{\text{test}}\right)=\exp\left\{-\frac{\sum_{T\in C_{\text{test}}}\log\;p\left(T\right)}{\sum_{i=1}^{\left|C_{\text{test}}\right|}N_{i}}\right\}. \end{array}$$

Here, the denominator in formula (9) represents the total length of the test set, *p*(*T*) in the numerator represents the probability of each word in the test set, and the specific calculation formula of *p*(*T*) is as follows:

(10) $$\begin{array}{c} p\left(T\right)=p\left(Z|D\right)*p\left(T|Z\right). \end{array}$$

Here, *p*(*Z|D*) represents the probability of each topic in a document, and *p*(*T|Z*) represents the probability of each word in a certain topic. In the following experiments, the Perplexity indicator is abbreviated as PERP.

To some extent, the evaluation of topic models by perplexity is essentially achieved by evaluating the performance of the model in downstream tasks, so this is an indirect method. Actually, there are some direct evaluation methods that are mainly based on the internal characteristics of the language. “Topic coherence” is another type of evaluation method used in this paper. This type of method is mainly used to automatically reveal the coherence of topic, where the larger the coherence value, the better the topic model. Its basic idea is rooted in the *distribution hypothesis of linguistics*, and many calculation methods such as *C*_*U* Mass_, *C*_*UCI*_, and *C*_*v*_ have been proposed based on this hypothesis [39]. In literature [40], Röder et al. systematically explored numerous topic coherence measures and compared with available human topic ranking data, and finally found that *C*_*v*_ performs better. Therefore, this paper will adopt PERP and *C*_*v*_ to comprehensively evaluate the quality of topic model from an indirect and direct perspective.

#### 5.2.2. Topic Recognition

Topic recognition for news text can be considered as a classification problem for the long text. Considering that this module pays more attention to the quality of classification, this paper will use the common confusion matrix. For the news dataset in this paper, there are many categories. Correspondingly, for the single label multi-classification problem, Micro-F1 score is used to evaluate the proposed model:

(11) $$\begin{array}{c} \text{Micro}-\text{Precision}=\frac{\sum_{i=1}^{n}TP_{i}}{\sum_{i=1}^{n}TP_{i}+\sum_{i=1}^{n}FP_{i}},\\ \text{Micro}-\text{Recall}=\frac{\sum_{i=1}^{n}TP_{i}}{\sum_{i=1}^{n}TP_{i}+\sum_{i=1}^{n}FN_{i}},\\ \text{Micro}-F1=\frac{2\times \text{Micro}-\text{Precision}\times \text{Micro}-\text{Recall}}{\text{Micro}-\text{Precision}+\text{Micro}-\text{Recall}}. \end{array}$$

### 5.3. Experimental Results and Analysis

In the following experiments, we will first verify the effectiveness of the idea of fusion of the word embedding model and topic model for news topic recognition, and then explore the best way of fusion. Furthermore, we have reproduced some related research work in recent years, and finally verify the superiority of the proposed text topic recognition framework based on word embedding enhancement.

#### 5.3.1. The Effectiveness of Word Embedding Enhancement

Based on the theoretical analysis of different text representation methods (refer to Section 1), this paper proposes that the effective combination of topic model and word embedding model can enrich the text representation and benefit NLP downstream tasks. Existing researches have carried out some explorations around this idea, but there is still no fusion standard in the field of text topic recognition. At the same time, these works have not considered the fusion between the topic distribution of different granularities and the word embedding information. To solve the above problems, this paper further proposes a novel text representation method based on word embedding enhancement, and applies it to the feature extraction layer of the proposed news topic recognition framework. In order to verify the effectiveness of the proposed model and explore the impact of different fusion strategies on the results, we will set the following baselines including TF-IDF, LDA, Word2vec, Glove, SGL, CGL, SWL, and CWL (for convenience to differ from the experiment in Section 5.3.2, the output of LDA used in this section is the document-level topic distribution). The last four comparison models are described as follows, and the essence of them is to combine the word embedding model and the LDA model with different fusion strategies. As shown in Figure 4, it illustrates the meanings of two symbols “⊙” and “⊕” related to the fusion strategies involved in this paper:

1. SGL. Performing a vector summation operation on the text representations obtained by the Glove and LDA methods
2. CGL. Concatenating the representation vectors obtained by Glove and LDA methods
3. SWL. Performing a vector summation operation on the text representations obtained by the Word2vec and LDA methods
4. CWL. Concatenating the representation vectors obtained by Word2vec and LDA methods

The detailed experimental results are shown in Table 4. In addition to the model fusion strategy, we also focus on the influence of vector dimensions on the experimental results. It is necessary to point out that the vector dimension of text representation based on the topic model is equal to that based on the word embedding model under the fusion strategy. For Word2vec and Glove, we trained word embedding models with the output vector dimensions of 100, 200, 300, 400, and 500. Correspondingly, we also trained LDA models with equivalent topic number. The final topic recognition effect is positively correlated with the value of Micro-F1.

In general, the highest Micro-F1 value on the 20NewsGroup dataset does not exceed 0.83, which is related to factors such as the variety of topics in the dataset and the high similarity of some topics. From the perspective of the classifier, the results show that the effect of SVM is better than that of LR, which is consistent with the theoretical analysis results. From the perspective of the dimension of the text representation vector, it can be found that Micro-F1 is increasing with the increase of the dimension, but the growth rate gradually decreases. Especially for SWL and Word2vec models, when the dimension of vector is greater than 400, Micro-F1 basically remains unchanged or even decreases. In summary, the combination effect of the topic model and the word embedding model is obviously better than any single model, which shows the correctness of the conjecture that “the effective combination of the topic model and the word embedding model can enrich the text representation and then improve the NLP downstream task effect” to a certain extent. Among the above models, the CGL model performs the best, which denotes that the concatenation of representation vectors obtained by Glove and LDA can indeed enrich text representation information and improve the topic recognition quality.

Moreover, we analyze the quality of the text representation vector from a semantic perspective. In the semantic space, each document is represented as a dense vector. Assuming all documents are mapped into a 2-dimensional space, the densely distributed area indicates that the potential topics of these documents are relatively similar. Considering that the text representation vector has high-dimensional sparse characteristics, we use Uniform Manifold Approximation and Projection for Dimension Reduction (UMAP) [41] and K-means [42] for further analysis.

Figure 5 shows the results of semantic embedding based on the 20NewsGroup dataset. Within the four subgraphs, the color of points with similar semantic distance is consistent, which demonstrates that the corresponding text representation method has captured certain features in the semantic space. From TF-IDF to CGL model, the regional distribution of different colors is becoming more uniform and there are fewer isolated points and groups, which correspond to the category distribution of the 20NewsGroup. In summary, it can also be concluded that the word embedding enhancement can indeed enrich the semantic information of text representation.

#### 5.3.2. Comparison of the Proposed Topic Recognition Framework and Other Methods

In this section, comparative experiments will be carried out to verify the superiority of the proposed framework for the problem of news topic recognition. The relevant information of baselines is described as follows. Note that differing from the existing methods, this framework also considers the impact of the optimal number of topics on the final results. In order to make the experimental results more convincing, the word vector dimension and the LDA topic representation vector dimension in baselines are both set to 300:

1. FPW. Zhou et al. [11] proposed the combination of word embedding technology Word2vec, feature weighting technology TF-IDF, and the topic model LDA, which not only increased the expressive ability of the vector space model but also reduced the dimension. Meanwhile, this paper also proposes **FP2**, **FPC** models with different fusion strategies.
2. DRIWL. Wang et al. [7] proposed a more comprehensive document representation method based on Word2vec and LDA. This method uses the Euclidean distance between the topic vector and document embedding vector as the new text representation, which can not only make full use of the statistical relationship between document and topic but also consider the semantic information between words.
3. TDE. Hui et al. [43] proposed a text clustering method based on topic document embedding. The key of this method is to use LDA and the TF-IDF model to extend the Skip-Gram model, and finally achieve text-level topic document embedding. It inherits the ability of Skip-Gram model to capture the syntactic and semantic relationship between words, and also inherits the ability to distinguish various semantics of polysemous words and homophones.

From the perspective of model construction, all models in baselines improve the quality of text representation by making comprehensive use of the advantages of TF-IDF, LDA, Word2vec, and Glove. In this regard, we have conducted some analysis on all models involved in the experiment. The overview of different fusion models is revealed in Table 5, which shows the submodels involved in each model and the dimensions of the final obtained text representation vector with this model.

For the two text representation models proposed in this paper, it can be seen that the essential difference lies in the presentation granularity of the topic distribution, and the topic distribution dimension is related to *τ*, which means the number of topics when training the LDA model. Moreover, the parameter *τ* will affect the quality of the topic model, and then indirectly affect the quality of the whole framework. Therefore, it is necessary to explore the optimal number of topics before evaluating the proposed two representation methods.

For the 20NewsGroup dataset, some previous work pointed out that the optimal number of topics is around 20 [10]. For this reason, we selected some values from 10 to 30 as the number of topics to train the LDA model. The related evaluation indicators include PERP and *C*_*v*_. The specific experimental results are shown in Table 6.

For the above experimental values, we mark the best three results under different evaluation indicators. It can be found that when *τ* is set to 20, the results under the PERP and *C*_*v*_ indicators are better, which indicates that the topic quality and topic coherence generated by LDA are both relatively good. Finally, we choose *τ*=20 as the optimal topic number. Comprehensive analysis shows that when *τ* is set to 20, the quality of the LDA model obtained is better.

Figure 6 shows the Micro-F1 scores of different models on the test data. First of all, it is certain that the DTE and WTE models proposed in this paper are better. In addition, based on DTE and SVM, we can get the best recognition result. However, some models in the baseline use LDA, Word2vec, and TF-IDF at the same time. In general, such models are more complex and the target representation vector has a larger dimension, but this fusion method does not necessarily get a better topic recognition effect. Therefore, it can be shown that the concatenation of document-level topic representation and the Glove document embedding is a better method. Moreover, for the models in the baseline, we replace the Word2vec with Glove to add some comparison models. It can be found that the recognition equality of FPW^*∗*^, FPC^*∗*^, FP2^*∗*^, and TDE^*∗*^ on the test dataset is worse than that of FPW, FPC, FP2, and TDE. However, the recognition equality of DRIWL^*∗*^ is better than DRIWL. The primary reason is that the fusion effect of TF-IDF and Word2vec is better than the fusion effect of TF-IDF and Glove. Finally, to evaluate the above models from the perspective of the classifier, it can be found that SVM often has a better result than LR for topic recognition on this dataset.

Similarly, for the BBC News dataset, we set the number of topics between 5 and 55 to train the LDA model, and the detailed results are shown in Table 7.

For BBC News dataset, it is relatively small, so the training time of the LDA model has been significantly reduced. According to the results in Table 7, it can be found that the LDA model achieves the best results under the PERP and *C*_*v*_ when *τ*=20. Based on above analysis, we finally choose 20 as the optimal topic number. Then, we conducted corresponding comparative experiments, the results of which shown in Figure 7.

On the whole, SVM and LR classifiers both have achieved relatively high Micro-F1 results, which may due to the fact that the BBC News dataset has a small scale and few topic categories. Compared with other methods, the text representation obtained by the DTE method has a small dimension but performs the best, reaching 0.969 based on both SVM and LR classifiers. In contrast, the WTE text representation model has an average performance on this dataset, but the difference between results is no more than 0.1.

### 5.4. Discussion

Based on the idea that adding word embedding information on the basis of the topic model can enrich the semantic information of the document, we propose two granularity text representation models, which are named DTE and WTE. Both models perform unsupervised learning on corpus to obtain the final representation vectors, which is simple to implement and can improve the quality of text representation. After testing on different datasets with other models, we found the two models that have achieved better topic recognition results; especially, the DTE method achieves the highest Micro-F1 score by using different classifiers on different datasets. According to the above theoretical analysis and the subsequent experimental results, we have reason to believe that the effective combination of the topic model and the word embedding model can make up for the defects of a single model to a certain extent. At the same time, it also shows the effectiveness and superiority of the proposed method based on word embedding enhancement for the problem of news topic recognition.

For the above experiments, we can also draw some other conclusions. First of all, for the document-level topic distribution in the DTE method, it does not need to be large. For example, when the dimension of the representation vector is 600 with the CGL method on 20NewsGroup, it obtains the Micro-F1 scores of 0.812 and 0.796 based on SVM and LR, respectively. In Section 5.3.2, the DTE method obtains Micro-F1 scores of 0.810 and 0.799, respectively, with the representation vector of 320. Secondly, for models that use both the TF-IDF feature weight and word embedding technologies, the combination effect of TF-IDF and Word2vec is better than that of TF-IDF and Glove. This can be reflected in the test datasets of 20NewsGroup and BBC News in Section 5.3.2.

## 6. Conclusion

With the evolution of the big data era, we are facing more and more serious information load problems in real life. This paper aims to realize the accurate and automatic sorting of Internet news text data. Considering that the single topic model and the word embedding model have certain defects, and the fusion of the two can enrich the representation information of the text, we proposed a novel text representation method and conducted preliminary exploration based on the classic TF-IDF, LDA, Word2VEC, and Glove models. Finally, we proposed two granularity fusion strategies for the topic model and the word embedding model, named DTE and WTE. Besides, we also formed a topic recognition framework based on word embedding enhancement. The core of the framework is to achieve a better integration of topic distribution representation and word embedding information. And, its essence lies in the realization of a more informative text representation method, which not only considers the relationship between document and topic but also integrates the context information of words. Through a large number of experiments on the 20Newsgroup and BBC News datasets, we first verified that the combination of the topic model and the word embedding model can effectively take advantage of the topic distribution, semantic knowledge, and syntactic relationship to achieve better text representation. In addition, we also compare DTE and WTE with the methods in related literature, and the results further prove the effectiveness and superiority of the proposed method for the problem of news topic recognition.

For the work of this paper, we believe that there are still the following directions that are worthy of further study:

1. The word embedding enhancement concept proposed in this paper is implemented in a simple and efficient way with good results, but the deeper integration ideas have not been considered. Therefore, we can start from the mathematical principles of the model and try to design a better fusion model to solve more NLP downstream tasks.
2. It is noteworthy that the amount of data used in the above experiments is limited. When processing the real massive news texts, the single machine environment is not enough to support subsequent storage, management, and analysis tasks. In response to this practical problem, we consider extending the proposed method to the Spark platform.
3. Compared with classical SVM, our team found that the Relevance Vector Machine (RVM) not only had a better classification performance on large document datasets [44] but also showed certain advantages in terms of prediction speed [45] and model robustness [46]. Therefore, introducing RVM into the topic recognition task of news text is also one of our next research directions.

## Figures and Tables

**Figure 1:** An example of document-topic distribution and topic-word distribution in LDA.

**Figure 2:** Architecture of DTE and WTE text representation models.

**Figure 3:** The architecture of news topic recognition framework.

**Figure 4:** The structure about summation “⊙” and concatenation “⊕” operations of representation vectors.

**Figure 5:** Different representation vectors of 20 news groups are embedded into 2-dimensions using UMAP.

**Figure 6:** The topic detection results of the 20NewsGroup for different methods by SVM and LR.

**Figure 7:** The topic detection results of BBC News for different methods by SVM and LR.

**Table 1:** The definition and description of symbols involved in this paper.

Symbol definition	Description
*N*_*i*_	The number of tokens in document *D*_*i*_
*V*	The vocabulary that including all words of corpus
*τ*	The number of topics when training the LDA model
TM	LDA model obtained by training on corpus
*ϕ*	The number of word vector dimension when training the word embedding model
EM	Word embedding model obtained by training on corpus
DTD_*i*_	Document-level topic distribution for document *D*_*i*_
WTD_*i*_	Word-level topic distribution for document *D*_*i*_
DTE_*i*_	Text representation based on word embedding model and doc-level topic distribution
WTE_*i*_	Text representation based on word embedding model and word-level topic distribution
*δ*	Dimension of document representation vector
*Z*	Topic distribution
⊕	Symbol that means concatenation operation of vectors
⊙	Symbol that means summation operation of vectors
*C*=*C*_train_∪*C*_test_	Corpus set *C* consists of training corpus *C*_train_ and test corpus *C*_test_

**Table 2:** The information of the 20NewsGroup dataset.

Topic category	Len	Size	Topic category	Len	Size
comp.graphics	163.0	973	rec.autos	126.3	990
comp.os.ms.windows.misc	160.6	985	rec.motorcycles	118.4	996
comp.sys.ibm.pc.hardware	116.7	982	rec.sport.baseball	131.2	994
comp.sys.mac.hardware	109.0	963	rec.sport.hockey	155.3	999
comp.windows.x	174.3	988	misc.forsale	95.1	975
talk.politics.misc	232.7	775	sci.crypt	189.6	991
talk.politics.guns	189.9	910	sci.electronics	121.8	984
talk.politics.mideast	269.4	940	sci.med	173.8	990
alt.atheism	183.0	799	sci.space	174.9	987
soc.religion.Christian	194.2	997	talk.religion.misc	192.1	628

**Table 3:** The information of the BBC news dataset.

Topic category	Len	Size
Tech	507.4	401
Business	334.2	510
Sport	336.3	511
Entertainment	337.7	386
Politics	461.2	417

**Table 4:** Results of the 20NewsGroup in 20 classes for 7532 texts by SVM and LR.

Model	Average 5-fold micro-F1 score of different dimensions														
	100			200			300			400			500		
	*δ*	SVM	LR	*δ*	SVM	LR	*δ*	SVM	LR	*δ*	SVM	LR	*δ*	SVM	LR
TF-IDF	100	0.373	0.372	200	0.48	0.475	300	0.586	0.580	400	0.637	0.631	500	0.671	0.663
LDA	100	0.686	0.682	200	0.692	0.689	300	0.712	0.711	400	0.715	0.714	500	0.721	0.723
Glove	100	0.724	0.710	200	0.767	0.754	300	0.784	0.771	400	0.794	0.780	500	0.799	0.788
SGL	100	0.745	0.732	200	0.779	0.767	300	0.792	0.780	400	0.807	0.794	500	0.813	0.802
CGL	200	**0.782**	0.772	400	**0.804**	**0.792**	600	**0.812**	**0.796**	800	**0.822**	**0.806**	1000	**0.826**	**0.813**
Word2vec	100	0.740	0.733	200	0.765	0.756	300	0.766	0.755	400	0.769	0.758	500	0.765	0.755
SWL	100	0.747	0.743	200	0.777	0.769	300	0.782	0.771	400	0.787	0.777	500	0.787	0.777
CWL	200	0.780	**0.776**	400	0.795	0.787	600	0.793	0.782	800	0.793	0.783	1000	0.796	0.785

Bold indicates that values are the optimal results.

**Table 5:** Overview of different fusion models.

Model	Dim	Submodels	Model	Dim	Submodels
FPW	300	TF-IDF, LDA, Word2vec	TDE	600	TF-IDF, LDA, Word2vec
FPW^*∗*^	300	TF-IDF, LDA, Glove	TDE^*∗*^	600	TF-IDF, LDA, Glove
FPC^*∗*^	600	TF-IDF, LDA, Word2vec	DRIWL	300	LDA, Word2vec
FPC^*∗*^	600	TF-IDF, LDA, Glove	DRIWL^*∗*^	300	LDA, Glove
FP2	300	TF-IDF, LDA, Word2vec	DTE	300 + *τ*	LDA, Glove
FP2^*∗*^	300	TF-IDF, LDA, Glove	WTE	300 + *τ*	LDA, Glove

The upper right corner of the model with “^*∗*^” indicates that this model uses Glove as the word embedding model. And, the dim represents the dimension of the final document representation vector.

**Table 6:** The quality of the LDA model with different topic numbers based on the 20NewsGroup.

Evaluation indicators	Quality evaluation of LDA model under different topic numbers										
	10	15	17	18	19	20	21	22	23	25	30
PERP	**370.954**	371.873	**371.562**	371.723	372.899	**370.068**	371.960	377.523	389.457	388.428	395.543
*C*_*v*_	**0.498**	0.557	0.591	0.577	0.595	**0.621**	0.585	**0.608**	0.586	0.576	0.583

**Table 7:** The quality of the LDA model with different topic numbers based on BBC News.

Evaluation indicators	Quality evaluation of LDA model under different topic numbers										
	5	10	15	20	25	30	35	40	45	50	55
PERP	**246.258**	**247.429**	249.625	**245.917**	249.677	255.310	256.739	254.678	259.439	265.335	261.736
*C*_*v*_	0.448	**0.495**	0.478	**0.522**	0.454	0.445	**0.471**	0.462	0.469	0.442	0.462

For the above experimental values, we mark the best three results under different evaluation indicators.

## Data Availability

The data used to support the findings of this study are available from the corresponding author upon request.
